This article has been retracted.

# A Hybrid Algorithm of Ant Colony and Benders Decomposition for Large-Scale Mixed Integer Linear Programming

**DOI:** 10.1155/2022/1634995

**Published:** 2022-08-31

**Authors:** Tingting Shan, Zhaoxuan Qiu

**Affiliations:** School of Management, Nanjing University of Posts and Telecommunications, Nanjing 210003, China

## Abstract

The mixed integer linear programming (MILP) has been widely applied in many fields such as supply chain management and robot control, while how to develop a more efficient algorithm to solve large-scale MILP is still in discussion. This study addresses a hybrid algorithm of the ant colony and Benders decomposition to improve the efficiency. We firstly introduce the design of our algorithm, in which the Benders algorithm decomposes the MILP into a master problem and a slack problem, the ant colony algorithm generates initial solutions for the master problem, and heuristic rules obtain feasible solutions for the slack problem. Then, the computational experiments are carried out to verify efficiency, with a benchmark test and some medium-large scale examples. Compared with other algorithms like CPLEX, GUROBI, and traditional ACA, our algorithm shows a better performance with a 0.3%–4.0% optimality gap, as well as a significant decrease of 54.3% and 33.6% on average in the CPU time and iterations, respectively. Our contribution is to provide a low-workload, time-saving, and high-accuracy hybrid algorithm to solve MILP problems with a large amount of variables, which can be widely used in more commercial solvers and promote the utilization of the artificial intelligence.

## 1. Introduction

Mixed integer linear programming (MILP) is a highly complex combinatorial optimization problem that contains both variables and continuous variables [1], as well as an NP-complete problem [2]. Due to the multiple types of its decision variables, it has broad applications in solving managerial planning problems, such as supply chain management [3], robot control problems [4], and traffic flow problems [5, 6]. A general MILP model is shown as follows:

(1) $$\begin{array}{c} P\;\;\;Min\;\;\;z=cx+fy,\\ Ax\geq b,\\ Bx+Gy\geq d,\\ x\in Z_{+}^{n_{1}},y\in R_{+}^{n_{2}}. \end{array}$$

In Model 1, *z* denotes the value of the objective function of the MILP, which often stands for some minimized planning goal like the total cost or the distance of path; *x* and *y* are the decision vectors subject to linear inequality constraints and the requirements in a mixed integer linear programming model, and all the variables are positive; *n* is the total amount of the decision variables, including *n*_1_ integer variables and *n*_2_ continuous variables, *n* = *n*_1_ + *n*_2_; *m* is the amount of the constraints, including *m*_1_ constraints with only integer variables and *m*_2_ constraints with both integer and continuous variables, *m* = *m*_1_ + *m*_2_; *c* and *f* is the vector of the continuous type of coefficients of the integer decision vector *x* and the continuous decision vector *y*, respectively, and the number of the elements in each vector equals to the amount of each kind of variables, *c* ∈ *R*^*n*_1_^ and *f* ∈ *R*^*n*_2_^; the matrices *A*, *B*, and *G* contain the coefficients in the constraints, which is related to all the variables in pure integer constraints, the integer variables and the continuous ones in mixed constraints, respectively. *A* ∈ *R*^*m*_1_×*n*_1_^, *B* ∈ *R*^*m*_2_×*n*_1_^, *G* ∈ *R*^*m*_2_×*n*_2_^; *b* and *d* are the vectors including the constraint values,  *b* ∈ *R*^*m*_1_^ and *d* ∈ *R*^*m*_2_^. If *n*_1_ = *n* (*n*_2_ = 0), the problem is a pure integer linear program; if *x_i_*  ∈ {0,1}, ∀*I*, the problem is a binary (0-1) integer program; if *n*_2_ ≥ 1, the problem is a MILP problem.

Though MILP has a great significance in several managerial and computational contexts, there is a problem: the size of the MILP expands exponentially with the dimension of the decision variables; that is, the more the decision variables in the model, the more difficult it for the algorithm to run and work in CPU efficiently. When solving large-scale MILP problems, traditional algorithms will be hard to match the requirement of running in commercial solvers, which can be an obstacle of spreading the MILP model to the daily practices. Therefore, how to develop a more efficient algorithm to solve large-scale MILP problems is still in discussion in the academic community.

To deal with this difficulty, previous research focused on three algorithms, i.e., decomposition algorithm, evolutionary algorithm, and hybrid algorithm. The decomposition algorithm is to decompose a MILP into an original problem and a slack problem, such as Benders decomposition [7–10], column generation [11–15], and Lagrangian decomposition [16–18]. The evolutionary algorithm solves a MILP in accordance with evolutionary rules [19–25]. However, both decomposition and evolutionary algorithm have their unique shortcomings in the calculation. To make use of the advantages of more than two algorithms and avoid all the drawbacks, the hybrid algorithm is proposed to solve MILP problems [26, 27].

Our contributions include: (1) combining the both sides of advantages, we come up with a new hybrid algorithm based on the Benders decomposition with the ant colony algorithm and heuristic algorithm, which gives a new perspective to solving MILP in a special context of large-scale variables in an efficient way, trying to fill a research gap in developing a more efficient hybrid algorithm for large-scale MILP; (2) as our hybrid algorithm has excellent performances compared to other traditional algorithms, it can provide a low-workload, time-saving, and high-accuracy way to solve large-scale MILP problems in several managerial and computational contexts such as the logistics network management. As the requirement for the function of CPU is reduced, the cost paid in high-quality computing equipment will decrease significantly and thus the MILP can be widely used in more commercial solvers and significantly promote the utilization of the artificial intelligence in more and more parts of the life and production process.

Our paper is organized as follows: in Section 2, we review the literature relevant to our study. In Section 3, we introduce the solution procedure of the proposed hybrid algorithm. In Section 4, we carry out numerical experiments and report numerical results. In Section 5, we summarize the conclusions.

## 2. Literature Review

This study focuses on proposing a solution algorithm for MILP. The related research problems include the Benders decomposition algorithm, the hybrid algorithm of Benders decomposition, and evolutionary algorithms.

The Benders decomposition algorithm refers to decomposing MILP into an original problem and a slack problem to improve the computational speed. Existing research has analysed the performance of Benders decomposition to solve MILP through solution time, iteration number, and degree of acceleration. Poojari and Beasley compare Benders decomposition with a standalone solver (CPLEX) and benders decomposition using a genetic algorithm [9]. Fischetti et al. prove that Benders decomposition allows for a significant boost in the performance of a mixed integer programming solver [28]. Víctor et al. use Benders decomposition to solve the coverage problem of network-oriented design [29]. François et al. use benders decomposition to solve the two-dimensional packing problem [30]. For the robot cell scheduling problem, Komari Alaei et al. prove that the Benders decomposition algorithm can improve the efficiency of scheduling [31]. Kergosiena et al. propose a Benders decomposition-based heuristic that makes it possible to find feasible solutions and lower bounds in a production and outbound distribution scheduling problem with strict delivery constraints [32]. However, the general Benders decomposition algorithm has a drawback as well. It takes a long time to calculate the optimal solution even in an infinite loop. Based on this situation, Boland et al. present a heuristic approach to two-stage mixed integer linear stochastic programming models with continuous second-stage variables [33]. In addition, to improve computation efficiency, the authors investigate the use of proximity search as a tactical tool to drive Benders decomposition. The Benders decomposition algorithm can effectively solve medium-large scale problems. Lin et al. propose a heuristic implementation of the Benders decomposition method that routes additional single and multiple flows without resolving the routing problem [34]. Previous studies have shown that the proposed hybrid algorithm is superior in convergence rate, CPU time, and iteration number.

The hybrid algorithm incorporates evolutionary algorithm and heuristic rules into the benders decomposition framework. For the former, Awad et al. propose a mixed Benders decomposition approach with the ant colony optimization technique to solve a transfer line balancing problem [35]. This hybrid algorithm can get an optimal solution in a short time for the transfer line balancing medium-large scale problems. Ma and Zhang use multiobjective evolutionary algorithms to reveal the cost-efficiency balance of human brain networks [36]. Su et al. propose a multiobjective evolutionary algorithm for the detection of large-scale complex network communities [37]. For the letter, Osman and Baki propose a heuristic algorithm based on column generation to solve the vehicle routing problem with time windows [38]. Comparing the general benders decomposition with benders decomposition using a genetic algorithm, the hybrid algorithm is better than the general benders decomposition in terms of computational efficiency [9]. Liu and Dessouky propose a decomposition-based hybrid heuristic algorithm to solve the joint passenger and freight train scheduling problem [39].

## 3. Hybrid Algorithm of Ant Colony and Benders Decomposition

### 3.1. Basic Benders Decomposition

Benders decomposition algorithm provides a basic framework to solve MILP through decomposing the original complex problem into two problems, i.e., an original problem and a slack problem. The original problem and the slack problem could be solved in turn through the transmission of information [40]. Model 1 contains two decision problems, defined by integer decision variables *x* and continuous variables *y*, respectively. In this paper, the optimization on *x* is defined as the original problem or “master problem” (denoted as *P*_*M*_), and *y* is defined as a slack problem (denoted as *P*_*S*_). The slack problem can be written as follows:

(2) $$\begin{array}{c} P_{S}\text{Min }z=c\hat{x}+fy,\\ Gy\geq d-B\hat{x},\\ y\in R_{+}^{n_{2}}. \end{array}$$

In Model 2, *z* is the objective function value of the *P*_*S*_; $\hat{\text{x}}$ denotes a feasible solution of *x*. When solving the slack problem *P*_*S*_, $\hat{\text{x}}$ can be treated as a constant vector temporarily. Therefore, the dual problem of model 2, denoted as *P*_*D*_, can be obtained as follows:

(3) $$\begin{array}{c} P_{D}\text{Max }z_{1}={\bar{\pi }}^{T}\left(d-B\hat{x}\right),\\ {\bar{\pi }}^{T}G\leq f,\\ \pi \geq 0. \end{array}$$

In Model 3,  *z*_1_ denotes the objective function value of the *P*_*D*_, which will equal to z only when both of them reach the optimal value; *π* denotes the dual variables of the *P*_*S*_. That means we can transfer *P*_*S*_ into a standard form of a general linear programming problem like *P*_*D*_ and then the optimal *y* will be easily solved.

There are three possible solutions with respect to *P*_*S*_: (1) infeasible, then exit; (2) unbounded, in which case choose any unbounded extreme ray (denoted as ${\bar{\pi }}^{T}$) and add a feasibility cut ${\bar{\pi }}^{T}\left(d-Bx\right)\leq 0$ into the original problem. Since we need the minimum of *z* in the *P*_*S*_, the feasible cut can be seen as the upper limit of the objective function value of the *P*_*S*_; (3) bounded, in which case take an optimal solution (denoted as ${\tilde{\pi }}^{T}$) and add an optimality cut ${\tilde{\pi }}^{T}\left(d-Bx\right)\leq \theta$ into the original problem. Due to the same reason in the unbounded solution, the optimality cut will be treated as the lower limit of the objective function value of the *P*_*S*_.

Therefore, the original problem of Model 4, denoted as *P*_*M*_, can be written as follows:

(4) $$\begin{array}{c} P_{M}\text{Min }w=cx+\theta ,\\ Ax\geq b,\\ 0\geq {\tilde{\pi }}_{O}^{T}\left(d-Bx\right),\forall f=1,\ldots ,F,\\ \theta \geq {\tilde{\pi }}_{O}^{T}\left(d-Bx\right),\forall o=1,\ldots ,O,\\ x\in Z_{+}^{n_{1}},\theta \in R. \end{array}$$

In the *P*_*M*_, *w* denotes the final objective function value of MILP. θ is a variable of the master problem, *θ* = *fy* and the *y* is the optimal solution vector for all the continuous variables we gain by solving the *P*_*S*_. *F* and *O* denote the collection of feasibility cut and optimality cut, respectively. The procedures of Benders decomposition are shown as follows (Algorithm 1):

### 3.2. Hybrid Algorithm of Ant Colony Algorithm and Benders Decomposition

Medium-large scale MILP indicates it has a tremendous number of decision variables, which makes MILP more complicated and difficult to solve. Benders decomposition gives a framework to reduce the problem size, but it cannot guarantee the solution speed and convergence rate. To improve the solution speed of medium-large scale MILP, we propose a hybrid algorithm of the ant colony algorithm and Benders decomposition. It utilizes the ant colony algorithm to generate the initial solution for the master problem and uses a feasibility heuristic to get feasible solutions for the subproblem in each iteration. The hybrid algorithm flow chart is shown in Figure 1.

The ant colony algorithm is a kind of heuristic algorithm imitating ants' behavior. The idea is that a group of cooperating ants can find the shortest path between the nest and the food source. Ants achieve cooperation by leaving a certain amount of pheromone on the road. The pheromone left by an ant can be detected by other ants, and the more pheromones left on a road, the higher the probability of other ants will follow this path, and the path of the track will be more strengthened. The ant colony algorithm had been proposed for the MILP problems [41–43].

For the MILP in Model 1, there are *n*1+*n*2, decision variables. We regard each solution of each decision variable as a node. The ants select a node which is a current value for each variable. Therefore, after *n*1+*n*2 times, it can obtain a solution for MILP. The solution procedures of the hybrid algorithm of the ant colony algorithm and Benders decomposition are explained as follows:

Step 1: *Initialization*. Let *m* denote the number of the ant colonies. Therefore, it can generate *m* solutions according to Model 1. In each iteration, the newly updated pheromone concentration can be calculated as follows:
  (5) $$\begin{array}{c} \tau_{mn}^{\text{new}}=\rho \tau_{mn}^{\text{old}}+\frac{Q}{f_{\text{min}}}, \end{array}$$
where *τ*_*mn*_^new^ denotes the pheromone concentration of *m*^th^ ant in *n*^th^ variable in the current iteration,*τ*_*mn*_^old^ denotes the pheromone concentration of *m*^th^ ant in *n*^th^ variable in the previous iteration, *ρ* represents the disappearance rate of pheromone, *Q* is a constant which equals to 10^4^ in this paper, *f*_min_ denotes the optimal value in the current iteration.
Step 2: *Fitness function*. The fitness function is defined by the object function and the number of solution violating the constraints according to Model 1. It is defined as follows:
  (6) $$\begin{array}{c} F_{f}=\lambda f+\left(1-\lambda \right)\kappa , \end{array}$$
where *F*_*f*_ denotes the fitness function, *λ* represents the proportion of each solution object value, *f* denotes the object value of each solution, *κ* denotes the number of solution violating the constraints.
Step 3: *Selection*. Choose an optimal solution for Model 1 in the current iteration and update this optimal solution for the next iteration. For the ant choosing which solution node for each decision variable, the selection probability of m^th^ ant in n^th^ variable *p*_*mn*_ is given by the following equation:
  (7) $$\begin{array}{c} p_{mn}=\left\{\begin{array}{cc} \frac{\tau_{mn}}{\sum_{n\in N}\tau_{mn}\sum }, & \forall m=1,2,\ldots ,m,\\ 0, & \text{otherwise.} \end{array}\right. \end{array}$$
Step 4: *Feasibility adjustment*. The generated initial solutions using the ant colony algorithm may not satisfy all the constraints in Model 4. There are two cases: the first one is feasible solutions if initial solutions satisfy all the constraints; the second one is infeasible solutions if initial solutions do not satisfy all the constraints. To guarantee the feasibility of the master problem, we propose a feasibility adjustment rule to solve Model 4. The solution idea is illustrated as follows.
Let *ξ* denotes the corresponding polyhedron of its LP relaxation for Model 4. The feasibility adjustment rule that obtains the feasible solution of the master problem can be constructed in the following:
  (8) $$\begin{array}{c} P_{FM}\text{Min }\alpha^{I}{\left|\left|x^{I+1}-x^{I}\right|\right|}^{2}+\left(1-\alpha^{I}\right)\left(cx^{I+1}+\theta \right),\\ x^{I},\theta \in \xi , \end{array}$$
where *α*^*I*^ is geometrically decreased with a fixed factor *μ* ∈(0,1), i.e., *α*^*I*+1^ = *μα*^*I*^ and *α*^0^ = [0, 1], *x*^*I*^ denotes the feasible integral solution in iteration *I*, and *I*=0 denotes the initial solution from ant colony algorithm output, and *I* >0 denotes the feasible solution from the feasibility heuristic in iteration *I* – 1. We set the original *α*^0^ to 1. In order to generate a feasible solution, the feasibility heuristic method is also used by other scholars [1, 44–47].

In general, the procedure of the hybrid algorithm of the ant colony algorithm and Benders decomposition is described as follows (Algorithm 2).

## 4. Computational Experiments

In this section, we present computational experiments to compare the efficiency and effectiveness of the proposed hybrid algorithm with the Benders decomposition algorithm and CPLEX solver. We adopt a mathematical model for the vehicle assignment and distribution problem in short supply to describe the general mixed integer linear programming. We use this model to test our proposed algorithm and report the numerical results from one small scale and six medium-large scale experiments, respectively. All the tests in this section were tested on a Lenovo Y400 with Intel Core i5-3230 M CPU, 2.60 GHz frequency, and 4 GB memory.

### 4.1. Vehicle Assignment and Distribution Problem

In our model formulation, we use *S* to denote the collection of all supply points, *D* denotes the collection of all demand points, and *N* denotes the collection of nodes. If node *i*, *j* ∈*S*, node *i* and *j* represent the distribution center, otherwise, node *i* and *j* represent the demand point. Let *c*_*ij*_ represent the time cost from note *i* to note *j*. Let *k* represents the vehicle number, respectively. Let *K* denote the collection of vehicles. We use *q*_*k*_ to represent the maximum loading capacity of the vehicle *k*. Let *Q*_*j*_ denote the material demand at demand point *j*. There are two types of decision variables in the whole rescue vehicle dispatch period. Let *x*_*ij*_^*k*^ represent the flow originating at node *i* and arriving at node *j*. *x*_*ij*_^*k*^ is a binary decision variable. Let *y*_*j*_^*k*^ represent the resource allocated to node *j* by vehicle *k*. The assumption that the total amount of rescue materials is less than the total amount of rescue materials at the demand point are used in this study and each vehicle cannot travel between supply points.

The mathematical model for the vehicle assignment and distribution problem in short supply can be rewritten by the following equation:

(9) $$\begin{array}{c} Min\;\;\;\sum_{i\in N}\sum_{j\in N}\sum_{k\in K}c_{ij}\cdot x_{ij}^{k}+\sum_{j\in N}\left(Q_{j}-\sum_{k\in K}y_{j}^{k}\right),\\ s.t.\sum_{i\in S}\sum_{j\in D}x_{ij}^{k}=1,\forall k\in K,\\ \sum_{i\in D}x_{ij}^{k}-\sum_{i\in D}x_{ji}^{k}=0,\forall j\in D,\forall k\in K,\\ \sum_{j\in N}x_{ij}^{k}\leq 1,\forall i\in D,\forall k\in K,\\ \sum_{k\in K}y_{j}^{k}\leq Q_{j},\forall j\in D,\\ \sum_{j\in D}y_{j}^{k}\leq q_{k},\forall k\in K,\\ y_{j}^{k}\leq Q_{j}\cdot \sum_{i\in N}x_{ij}^{k},\forall j\in D,\forall k\in K,\\ x_{ij}^{k}\in \left\{0,1\right\},y_{j}^{k}\in Z_{+}. \end{array}$$

where ∑_*i*∈*N*_∑_*j*∈*N*_∑_*k*∈*K*_*c*_*ij*_ · *x*_*ij*_^*k*^ denotes the total time cost of vehicles and ∑_*j*∈*N*_(*Q*_*j*_ − ∑_*k*∈*K*_*y*_*j*_^*k*^) denotes the total unmet material at demand points. In this optimization model, constraints 10∼12 are the flow conservation equations. Constraint 13 states that the quantity of materials released is smaller or equal to the quantity demand at each demand point. Constraint 14 ensures that the quantity of materials released is smaller and equal to its maximum load by each vehicle. Constraint 15 states the relationship between two variables. Finally, Constraint 16 ensures that *x*_*ij*_^*k*^ is a binary variable and *y*_*j*_^*k*^ is the positive integer variable.

### 4.2. Small Scale Experiment: A Benchmark Test

All parameter values are shown in this section. In the example, we assume that the number of supply point *S* is equal to 2, the number of demand point *D* is equal to 5, the number of vehicle *K* is equal to 3, and the material demand at demand points 1, 2, 3, 4, and 5 are 400, 500, 200, 600, and 300 separately, the maximum loading capacity of the vehicle 1, 2, and 3 are 800, 400, and 300, respectively, the time cost *c*_*ij*_ is shown in Table 1. Due to the assumption that each vehicle cannot travel between supply points, we cite a very large number *M* in Table 1.

The results using CPLEX (version 12.6), GUROBI, Benders decomposition, ADMM, ACA, and hybrid algorithm are shown in Table 2 and Figure 2, respectively. According to the results shown in Table 2, the CPU times of the small scale experiment using CPLEX, GUROBI, Benders decomposition, ADMM, ACA, and hybrid algorithm are 1.58 seconds, 1.21 seconds, 32.3 seconds, 0.39 seconds, 0.40 seconds, and 0.35 seconds, respectively. For one thing, our hybrid algorithm can save 99.8% of the CPU time in maximum compared with general Benders decomposition and 10.3% of the CPU time in minimum compared with ADMM, with an average decrease of 54.3%; for another, this algorithm can save 50% of the number of iterations in maximum compared with CPLEX and 14.3% of the number of iterations in minimum compared with ADMM, with an average decrease of 33.6%. Besides, we compare the upper bound, lower bound, CPU time, iteration number, and gap of six algorithms. The trend of the upper and lower bound for CPLEX, GUROBI, Benders decomposition, ADMM, ACA, and hybrid algorithm is shown in Figure 2. Obviously, the upper and lower bounds of six algorithms are equal in the 12^th^, 11^th^, ninth, eighth, seventh, and sixth iteration, respectively. Therefore, this result proves that the efficiency of the proposed hybrid algorithm is better than the other five algorithms. The accuracy of CPLEX, GUROBI, and general Benders decomposition algorithm are better than the proposed hybrid algorithm in this small scale experiment. The accuracy of the proposed hybrid algorithm is better than ADMM and ACA in this small scale experiment.

### 4.3. Medium-Large Scale Experiments: Further Comparison

In order to better compare the advantages and disadvantages of six algorithms in this paper, we expand the number of supply point, the number of vehicle, and the number of demand point based on a benchmark example. Meanwhile, we expand other parameters in the model. There are 9 cases of medium-large scale experiments in the paper. We set the small scale experiment as Case 1. The numerical results of medium-large scale numerical examples that are solved by CPLEX, GUROBI, Benders decomposition, ADMM, ACA, and hybrid algorithm are recorded in Tables3 and 4. The total physical nodes of the vehicle assignment and distribution network in the nine medium-large scale cases are 20, 25, 30, 35, 35, 40, 45, 50, and 60, respectively. Therefore, the total variable size of the vehicle assignment and distribution network in the nine medium-large scale cases are 1175, 2075, 3225, 4600, 6450, 9200, 12500, 16300, and 30825, respectively.

We can obtain upper bound, lower bound, CPU time, and gap by CPLEX, GUROBI, Benders decomposition, ADMM, ACA, and hybrid algorithm. We report CPU time and iteration number amongst six algorithms for each case in Figures 3 and 4, respectively. In order to better reflect the relationship between CPU time data, we do the followings: (1) divide the CPU time greater than 300 by 10 in Figure 3; (2) we set the CPU time for Case 10 by CPLEX and GUROBI equal to 5000 in Figure 3; (3) due to the CPU time of Benders decomposition is too long, we set a maximum time point to 3600 seconds. In order to better reflect the relationship between iteration number data, we do the following: set the iteration number for Case 10 by CPLEX and GUROBI equal to 150 in Figure 4. From the results of nine medium-large scale experiments, the calculation accuracy and calculation time are the same as that of small scale experiment. That is because Benders decomposition solves the master problem by using a function named CPLEXMILP in each iteration. The master problem has more and more cuts. Therefore, the running time of general Benders decomposition is longer than other algorithms for each example, which is not an appropriate technique if we solve the MILP problem with a commercial solver.

Summarily, compared to the Benders decomposition, ADMM, and ACA, the hybrid algorithm has better computational efficiency. The hybrid algorithm has better computational accuracy than ADMM and ACA in this paper. Obviously, the hybrid algorithm is more suitable for the MILP problem than CPLEX, GUROBI, Benders decomposition, ADMM, and ACA.

## 5. Conclusions

This study focuses on proposing a new hybrid algorithm that contains ant colony and feasible heuristic decomposition with consideration of solving the large-scale MILP problems with higher computing efficiency. Firstly, we have used the ant colony algorithm and heuristic rules to calculate the initial and feasible solution for the master and slack problem, respectively, gaining the initial elements that are more approaching to the optimal solution of the MILP to speed up the Benders computing process. Subsequently, using vehicle assignment and distribution problem as a background, our hybrid algorithm has been applied in a series of computational experiments to verify its efficiency. The numerical results in the benchmark test have demonstrated that our hybrid algorithm significantly saves about 54.3% and 33.6% on average in the CPU time and iterations, respectively. Compared with other algorithms, our hybrid algorithm shows the superiority of computational performance with only 43.20s of CPU time, a 2.6% gap even in the largest 60-node example, which means our algorithm is always the fastest one and required the least iterations with a high robustness.

Our research also has some limitations, which could pave the fruitful path for the future works. Firstly, the major limitation is that we only focus on extending the application of the Benders decomposition with ant colony in solving large-scale MILP problems in the reality due to the advantages indicated by previous studies. Besides, inefficiency may occur in coincidence when dealing with some data with very special structure due to the limitation of the random search technique applied in many heuristic algorithm. For future studies, more traditional algorithms such as CPLEX or GUROBI, etc., can be taken into consideration to improve the efficiency of other large-scale programming problems. Scholars can explore more new hybrid algorithms with other excellent metaheuristic algorithms, especially to avoid the coincident inefficiency when processing some special data, or develop new ways to deal with large-scale problems in the context of the Big Data epoch in the future.

## Figures and Tables

**Figure 1:** The flow chart of hybrid algorithm.

**Figure 2:** The trend of the upper and lower bound.

**Figure 3:** CPU time amongst three algorithms for each case.

**Figure 4:** Iteration number amongst three algorithms for each case.

**Algorithm 1:** Procedures of benders decomposition.

**Algorithm 2:** Procedures of hybrid algorithm of ant colony algorithm and benders decomposition.

**Table 1:** Temperature and wildlife count in the three areas covered by the study.

	*S* = 1	*S* = 2	*D* = 1	*D* = 2	*D* = 3	*D* = 4	*D* = 5
*S* = 1	*M*	*M*	12	15	9	6	24
*S* = 2	*M*	*M*	11	8	12	13	4
*D* = 1	12	11	*M*	18	6	16	9
*D* = 2	15	8	18	*M*	15	20	11
*D* = 3	9	12	6	15	*M*	17	14
*D* = 4	6	13	16	20	17	*M*	11
*D* = 5	24	4	9	11	14	11	*M*

**Table 2:** Numerical results of benchmark example.

Approach	Upper bound	Lower bound	CPU (s)	Iteration	Gap (%)
CPLEX	544	544	1.58	12	0
GUROBI	544	544	1.21	11	0
Benders	544	544	32.3	9	0
ADMM	590	531	0.39	8	8.2
ACA	602	527	0.40	7	10.6
Hybrid algorithm	586	537	0.35	6	4

**Table 3:** Numerical results of medium-large scale numerical examples.

Parameters			Variable size		CPLEX				GUROBI				Benders decomposition			
*S*	*D*	*K*	*x*	*y*	UB	LB	CPU (s)	Gap (%)	UB	LB	CPU (s)	Gap (%)	UB	LB	CPU (s)	Gap (%)
2	5	3	147	15	544	544	1.58	0	544	544	1.21	0	544	544	32.3	0
5	10	5	1125	50	3257	3257	3.20	0	3257	3257	2.81	0	3257	3257	102	0
5	15	5	2000	75	4313	4313	4.60	0	4313	4313	3.98	0	4313	4313	134.0	0
5	20	5	3125	100	6777	6777	5.66	0	6777	6777	4.23	0	6777	6777	156.0	0
10	20	5	4500	100	7051	7051	6.05	0	7051	7051	5.58	0	7051	7051	196.0	0
5	20	10	6250	200	7886	7886	6.84	0	7886	7886	5.92	0	7886	7886	275.0	0
10	20	10	9000	200	8008	8008	7.32	0	8008	8008	6.59	0	8008	8008	365.0	0
10	25	10	12250	250	8117	8117	351	0	8117	8117	235	0	8117	8117	1221.0	0
10	30	10	16000	300	10307	10307	2524	0	10307	10307	2012	0	14270	10001	3600.0	38
15	30	15	30375	450	—	—	—	—	—	—	—	—	34407	9853	3600.0	145

**Table 4:** Numerical results of medium-large scale numerical examples.

Parameters			Variable size		ADMM				ACA				Hybrid algorithm			
*S*	*D*	*K*	*x*	*y*	UB	LB	CPU (s)	Gap (%)	UB	LB	CPU (s)	Gap (%)	UB	LB	CPU (s)	Gap (%)
2	5	3	147	15	590	531	0.39	8.2	602	527	0.40	10.6	586	537	0.35	4.0
5	10	5	1125	50	3302	3214	1.80	1.4	3314	3201	1.80	1.7	3298	3231	1.70	0.7
5	15	5	2000	75	4395	4287	2.50	1.9	4420	4239	2.60	2.4	4327	4306	2.40	0.3
5	20	5	3125	100	6890	6651	4.20	2.5	6999	6608	3.50	3.0	6814	6699	3.60	1.2
10	20	5	4500	100	7234	6901	3.90	6.2	7981	6681	3.90	8.3	7092	6990	3.80	0.5
5	20	10	6250	200	8016	7629	4.20	3.3	8210	7523	4.20	4.6	7901	7842	4.10	0.5
10	20	10	9000	200	8299	7893	5.20	4.6	8465	7768	5.60	5.7	8104	7962	4.90	1.2
10	25	10	12250	250	8207	8014	16.70	1.6	8287	7995	17.30	2.1	8186	8087	15.50	0.3
10	30	10	16000	300	11416	9960	21.30	8.4	11409	9893	20.30	10.6	10423	10167	19.70	1.4
15	30	15	30375	450	14590	13027	46.70	6.3	15409	12580	49.30	10.1	14407	13664	43.20	2.6

## Data Availability

The data used to support the findings of this study are available from the corresponding author upon request.
